RETRACTED

# Psychological Changes of Social Media on Charitable Cultural Behavior Based on Big Data Technology

**DOI:** 10.1155/2022/5871669

**Published:** 2022-08-20

**Authors:** Xi Chen

**Affiliations:** School of Public Administration and Policy, Renmin University of China, Beijing 100872, China

## Abstract

With the advent of the era of big data, the world is facing the challenge of unprecedented information blowout growth, and Internet information processing technology has also ushered in rapid development. At the same time, charity culture has always been a part that the state and society attach great importance to. It is a form of social wealth redistribution and a supplement to the social security system. Based on this social background and reality, this paper analyzes and explores the psychological changes of charitable cultural behavior by social media based on big data technology. This paper introduces latent semantic analysis and constructs the theoretical framework of social media. This paper introduces the related concepts of heart rate variability and mental state, collects the factor factors and constructs the model, and studies the PLS load and cross load. This paper makes a statistical analysis of the data of charitable donations in China from 2017 to 2021 and tests the validity of the questionnaire from the psychological level. The experimental results show that the correlation between the subscales of the questionnaire and the total scale is between 0.470 and 0.820, and the correlation between the dimensions is between 0.183 and 0.590. The correlation between the dimensions and the total score of the scale is higher than that between the dimensions, which shows that there are both connections and differences between the dimensions of the two scales, which are relatively independent, and the scale has a certain structural validity.

## 1. Introduction

In the development process of psychological research, the psychological state has changed from the psychological basic theory to the psychological dimension theory, which is the complex and changeable psychological dimension theory of people's psychology. In order to accurately represent and evaluate people's mental state, it is necessary to establish an effective mental state model. According to the different judgment methods, the judgment of psychological state is mainly divided into two categories: judgment of nonphysiological signals and judgment of physiological signals. The mental state judgment based on nonphysiological signals is mainly judged by facial expressions and speech. Based on the above background, the main research content of this paper is to screen samples from the level of social media. It explores the analysis of psychological state changes on the topic of charitable cultural behavior. The innovations of this paper are as follows: (1) the CBOW model and the Skip-Gram model are reconstructed. In the projection layer, the two word vectors in the input layer are accumulated and summed, which greatly simplifies the algorithm. (2) The internal correlation coefficient analysis of latent variables was carried out, which made the discriminant validity more obvious. (3) The donations received by various types of entities in 2021 are selected as the second sample data, which is obviously convincing and time-sensitive.

RETRACTED

## 2. Related Work

Social media is an emerging social tool that is widely used around the world. Rothkrantz proposed a matching algorithm in teaching mode for creating peer groups to perform group work. In distance learning, students are remote in time and place. Social media can provide a virtual meeting place. But his research does not divide social media into mobile and host [1]. Christian surveyed the results of a survey of 1,034 citizens of 30 European countries between February and June 2015. It aims to explore citizens' attitudes towards the use of social media for private purposes and emergencies [2]. Allcott Gentzkow discussed the economics of fake news and provided new data on fake news consumption ahead of the election. A new online survey was conducted based on web browsing data, fact-checking website archives [3]. Enikolopov et al. conducted research to consider whether new media would promote accountability as a social and political topic in nondemocratic countries, where traditional media are often suppressed [4].

Subsequently, foreign academic and practical circles continued to discuss and study it. Management, economics, law, ethics, and many other schools of thought study corporate philanthropy from their respective fields. Charitable cultural behavior is a supplement to the social security system. Jeffery et al. argued that reduced access to farmland in the background and food insecurity in urban areas has expanded the need for emergency food aid. His research assessed the relationship between charitable food assistance clients' federal nutrition program use, local resources, and fresh produce consumption [5]. Research by Sneddon found that personal values influence charitable giving decisions. He aimed to emphasize that research on donor values can provide a more nuanced understanding of their motivations for choosing philanthropy. It also has the potential to inform the research and practice of fundraising. But he did not sort out the relationship between personal values and charitable giving [6]. Yang Y examined the intergenerational effects of individual charitable giving in China based on China's unique social structure, traditional culture, and philanthropic history. He identified the mutual influence of children's charitable giving and parental charitable giving through downward and upward intergenerational transmission. It is demonstrated that the effect of upward propagation is greater than that of downward propagation [7].

RETRACTED

## 3. Changes in Mental State

### 3.1. Latent Semantics in Big Data

The earliest citation of the term “big data” can be traced back to apache Org's open-source project Nutch. At that time, big data was used to describe a large number of data sets that needed batch processing or analysis to update the network search index. Latent Semantic Analysis performs statistical analysis of large amounts of text to extract the semantics of terms in the text. This semantic information is essentially the sum of contextual information in the text. Representing text and terms with semantic structure eliminates the correlation between terms and simplifies text vector representation [8]. With the development of various social networking sites and other emerging service industries, the type and scale of data in human society are growing rapidly, which marks that we have entered the era of big data.

LSA uses a term-text matrix to describe the relationship between text and terms. The term-text matrix is a sparse matrix where each row represents a term, and each column represents a text:

(1) $$\begin{array}{c} X=\left[\begin{array}{ccc} {\text{weight}}_{1,1} & \ldots & {\text{weight}}_{1,n}\\ \ldots & \ldots & \ldots \\ {\text{weight}}_{m,1} & \ldots & {\text{weight}}_{m,n} \end{array}\right]. \end{array}$$

Among them, the elements on the diagonal of matrix Σ are singular values. Left singular vectors form a matrix, and right singular vectors form a matrix:

(2) $$\begin{array}{c} X=U\times \Sigma \times V^{T}. \end{array}$$

The correlation matrix of terms and texts can be expressed as follows:

(3) $$\begin{array}{c} \begin{array}{c} XX^{T}=\left(U\Sigma V^{T}\right){\left(U\Sigma V^{T}\right)}^{T}=\left(U\Sigma V^{T}\right)\left(V^{T^{T}}\Sigma^{T}U^{T}\right)=U\Sigma \Sigma U^{T},\\ X^{T}X={\left(U\Sigma V^{T}\right)}^{T}\left(U\Sigma V^{T}\right)=\left(V^{T^{T}}\Sigma^{T}U^{T}\right)\left(U\Sigma V^{T}\right)=V\Sigma^{T}\Sigma V^{T}. \end{array} \end{array}$$

The correspondence between text, latent variables, and terms in the PLSA model is shown in Figure 1.

The joint probability formula [9] is defined for the modeling process:

(4) $$\begin{array}{c} p=\left(t_{i},w_{j}\right)=p\left(t_{i}\right)p\left(w_{j}|t_{i}\right), \end{array}$$

(5) $$\begin{array}{c} p\left(w_{j}|t_{i}\right)=\sum_{k=1}^{K}p\left(w_{j}|z_{k}\right)p\left(z_{k}|t_{i}\right). \end{array}$$

Using the Bayesian formula, formula (5) is transformed into the following formula:

(6) $$\begin{array}{c} p\left(t_{i},w_{j}\right)=\sum_{k=1}^{K}p\left(z_{k}\right)p\left(t_{i}|z_{k}\right)p\left(w_{j}|z_{k}\right). \end{array}$$

The likelihood function is found as follows:

(7) $$\begin{array}{c} L=\sum_{i=1}^{M}\sum_{j=1}^{N}n\left(t_{i},w_{i}\right)\log p\left(d_{i},w_{i}\right). \end{array}$$

The iterative process of the EM algorithm mainly includes *E* steps and *M* steps [10]:

(1) Step E: calculate the posterior probability of the latent variable by estimating the currently known parameters by the following formula:
  (8) $$\begin{array}{c} p\left(z_{k}|t_{i},w_{j}\right)=\frac{p\left(z_{k}\right)p\left(z_{k}|t_{i}\right)p\left(w_{j}|z_{k}\right)}{\sum_{l=1}^{k}p\left(z_{l}\right)p\left(z_{k}|t_{i}\right)p\left(w_{j}|z_{l}\right)}. \end{array}$$
(2) M step: the posterior probability calculated by the *E* step updates the probability distribution:
  (9) $$\begin{array}{c} p\left(w_{j}|z_{k}\right)=\frac{\sum_{i=1}^{m}n\left(t_{i}\cdot w_{j}\right)p\left(z_{k}|t_{i},w_{j}\right)}{\sum_{i=1}^{M}\sum_{l=1}^{N}n\left(t_{i},w_{l}\right)p\left(z_{l}\right)p\left(z_{k}|t_{i},w_{l}\right)}, \end{array}$$
  (10) $$\begin{array}{c} p\left(t_{i}|z_{k}\right)=\frac{\sum_{i=1}^{N}n\left(t_{i}\cdot w_{j}\right)p\left(z_{k}|t_{i},w_{j}\right)}{\sum_{i=1}^{M}\sum_{j=1}^{N}n\left(t_{i},w_{l}\right)p\left(z_{l}\right)p\left(z_{k}|t_{i},w_{l}\right)}, \end{array}$$
  (11) $$\begin{array}{c} p\left(z_{k}\right)=\frac{\sum_{l=1}^{M}\sum_{j=1}^{N}n\left(t_{i}\cdot w_{j}\right)p\left(z_{k}|t_{i},w_{j}\right)}{\sum_{l=1}^{M}\sum_{J=1}^{N}n\left(t_{i},w_{l}\right)}. \end{array}$$
E-step and M-step are continuously calculated interactively until the likelihood function reaches a maximum value.

First, get the joint generation probability of the entire document set:

(12) $$\begin{array}{c} p\left(w,z|\alpha ,\beta \right)=p\left(w|z,\beta \right). \end{array}$$

Through analysis, it can get

(13) $$\begin{array}{c} p\left(w|z,\beta \right)=\prod_{k=1}^{K}\prod_{k=1}p\left(w_{i}=t|z_{i}=k\right). \end{array}$$

Through analysis, it can get

(14) $$\begin{array}{c} p=\left(z|\theta \right)=\prod_{m=1}^{M}\prod_{k=1}^{K}\left(z=k|m\right). \end{array}$$

The joint probability distribution is obtained by (12)–(14):

(15) $$\begin{array}{c} p\left(w,z|\alpha ,\beta \right)=\prod_{k=1}^{K}\prod_{z_{i}=k}p\left(w_{i}=t|z_{i}=k\right)\times \prod_{m=1}^{M}\prod_{k=1}^{K}\left(z=k|m\right). \end{array}$$

Two probability distributions are introduced [11]:

Distribution A:

(16) $$\begin{array}{c} p\left(\text{nexttable}\right)=\text{occupied occupied }r_{j}|\text{previous }m-1,\gamma =\frac{n_{j}}{\gamma +m-1}, \end{array}$$

(17) $$\begin{array}{c} p\left(\text{nexttable}\right)=\text{occupied table}|\text{previous }m-1,\gamma =\frac{\gamma }{\gamma +m-1}. \end{array}$$

Machine learning algorithms cannot directly recognize text in natural language. Therefore, it is first necessary to convert the natural language into a form that the algorithm can recognize. Word vector is the product of mathematical processing of natural language [12].

(18) $$\begin{array}{c} \text{Vectors}\left(WC\right)=\left\{v^{\prime }=\left[\begin{array}{c} 1\\ 0\\ 0\\ 0\\ 0 \end{array}\right],v^{\text{like}}=\left[\begin{array}{c} 0\\ 1\\ 0\\ 0\\ 0 \end{array}\right],v^{\text{Twitter}}=\left[\begin{array}{c} 0\\ 0\\ 1\\ 0\\ 0 \end{array}\right],v^{\text{learning}}=\left[\begin{array}{c} 0\\ 0\\ 0\\ 0\\ 1 \end{array}\right]\right\}. \end{array}$$

RETRACTED

### 3.2. CBOW Model and Skip-Gram Model

The main function of CBOW is to predict words based on known words in the current context. The CBOW model mainly includes three layers: input layer, projection layer, and output layer. Suppose that there is a training sample Context(*w*), where *w* represents a word, and Context(*w*) represents the first *c* and last *c* words of word *w* [13], as shown in Figure 2.

In the projection layer, the 2 word vectors in the input layer are accumulated and summed. The formula is as follows:

(19) $$\begin{array}{c} X_{w}=\sum_{i=1}^{2c}v\left(\text{Context}\left(w\right)i\right). \end{array}$$

The Skip-Gram model predicts its context from a given word. Its model mainly includes three layers: input layer, projection layer, and output layer. Among them, the input layer is the word vector of words [14]. The maximum value of formula (20) is obtained by the projection layer:

(20) $$\begin{array}{c} \frac{1}{T}\sum_{t=1}^{T}\sum_{-c\leq j\leq c}\log p\left(W_{t+j}{|W}_{t}\right). \end{array}$$

### 3.3. Theoretical Framework

With the development and application of computer technology in social life, the growth rate of information is gradually accelerating, and the total amount of information is also rapidly increasing, which has led to changes in its form—quantitative change leads to qualitative change and has accumulated to a level sufficient to trigger change. The characteristics of big data can be summarized by four “Vs,” namely volume, variety, velocity, and value. Consent mobilization on social media can be summarized into three stages: cognitive construction, affective mobilization, and action mobilization. Through “speech content” and “emotional performance,” cognitive construction and emotional mobilization can be achieved in the audience, thereby constructing “meaning” and “identity.” This way, participants can act on their behalf and mobilize for action. However, consent mobilization on social media takes place in a virtual online world where both mobilizers and participants are hidden and decentralized. The power of this “discussion” and “consciousness” is mobilized differently and uncertainly in each “person.” The prediction of big data is based on the correlation analysis of massive data. The era of big data provides us with a new way of thinking. It is no longer keen on exploring the causal relationship between things, but to explore possible related things through correlation, replacing the traditional error prone methods based on assumptions.

RETRACTED

Research on the impact of consensus mobilization has primarily focused on the impact of mobilization information on individuals. It refers to the concept of “communicative effect” in communication, which refers to the changes in psychology, attitude, and behavior caused by persuasive communicative behavior. In communication, the effect of communication is divided into three levels: external information acts on people's perception and memory systems, causing people's knowledge growth and changes in cognitive structure, which belong to the influence of cognitive level. Effects on people's perceptions and value systems, as well as changes in emotions or feelings, are psychological and attitudinal effects. These changes are manifested in what people say and do; that is, they become the result of actions. In the communication effect, from cognition to attitude to action, it is a process of accumulation, deepening, and expansion of effect [15]. The communication effect of the former level also affects the communication effect of the latter level. The entire research model is shown in Figure 3.

The application of social media has attracted widespread attention at home and abroad, but in the practice of applying it to archival work, foreign archival circles precede China, and countries such as the United States and France have applied more social media in archival work.

### 3.4. Definition of Social Media Word of Mouth

The social responsibility concept of “putting the economic interests of enterprises first” no longer has a dominant position. People began to reexamine the social responsibility of enterprises, and it has become a common understanding that enterprises should bear other responsibilities than economic responsibility. Some academics define social media as “potential, actual, and former consumers' positive or negative perceptions of a product or company.” Some researchers also define it as “a virtual world where people can communicate their comments about a product or service by typing.” Social behaviors take many forms on the Internet, mainly including ratings, likes or dislikes, comments, recommendations, experience exchanges, and promotions. And through empirical research, it is proved that the socialized enterprise structure can be divided into three dimensions: recommendation and promotion, rating and comment, and forum and community. On this basis, the normative use of social media is created and empirically demonstrated that recommendation and promotion are important components.  Figure 4 shows the social media word-of-mouth research model [16].

RETRACTED

Social media was originally designed for socializing, not for consumers to shop. Therefore, the specific functional design is different from that of shopping websites, resulting in changes in the way consumers participate in word-of-mouth. The author believes that this change needs to be considered [17]. In terms of research areas, domestic research is mainly concentrated in the more developed regions in the southeast, and there is less research on enterprises in the northwest.

### 3.5. Heart Rate Variability

HRV refers to the difference in the interval between sustained heartbeats. The difference in heart rate interval is determined by the push from the sinoatrial node. The impulses from the sinoatrial node are determined by the activity of the sympathetic and parasympathetic nervous systems. Therefore, HRV is an indicator reflecting the activity and balance process of the autonomic nervous system. It can qualitatively and quantitatively evaluate autonomic function. Due to its advantages of rapidity, convenience, noninvasiveness, accuracy, and objectiveness, it has been widely used in clinical practice. It detects heart rate variability in patients with anxiety and depression. The study found that patients with anxiety and depression had reduced heart rate variability, indicating reduced autonomic nervous system function. Users who received negative news alerts on social media and other platforms were more likely to experience negative emotions such as anxiety and depression. Although they have lower levels than those with anxiety and depression, their heart rate variability can also be altered by psychological factors that can even lead to disturbances in the autonomic nervous system. At the same time, people have self-awareness and subjective evaluations of all aspects of themselves. Whether these knowledge and assessments are accurate and objective directly affects relevant thinking and behavior. Similarly, people also have subjective understanding and evaluation of their own psychological state. If the recognition and evaluation are scientific, accurate, and objective, these will have a good impact on philanthropic cultural behavior and social ethos. Conversely, if there is a deviation, there will be a negative impact on philanthropic cultural behavior and social style [18]. Negative words can reverse the emotional tendency of sentences and then change the emotional tendency of sentences.

RETRACTED

### 3.6. Negative Effects of Mental Subhealth State

“Mental subhealth” is an important type of subhealth. It is an intermediate state between mentally healthy and mentally unhealthy. These states all meet the psychiatric diagnostic criteria such as CCMD-III, ICO-10, and DSM-IV. But it has a great impact on people's life and work [19]. Through the self-rating scale, for example, if the self-perceived mental state persists for more than 2 weeks, the SCL-90 score is greater than 160, or the scores of each factor are greater than 2, the subjects are excluded from suspected psychosis or other mental diseases, that is, in a state of “mental subhealth” [20]. However, these studies tend to study natural symptoms, the most representative of which is the study of “chronic fatigue syndrome” in Western countries. The research on the classification of “ill-health” is still in its infancy.

### 3.7. Mental State Model

Benefits are not only economic benefits, but also political benefits. Through enterprise charity activities, entrepreneurs share the pressure of the government on some functions, so that the government has a good impression on the enterprise, and the enterprise owner can obtain a certain political identity, so as to create a good political environment for the enterprise.

At present, two-dimensional mental state classification models have been widely used. The first is to set the mental state in a polar coordinate system. The second is to label mental states based on enthusiasm and liking. Mental states are thus integrated into a two-dimensional Cartesian coordinate system. In the model, excitement and fatigue correspond to each other. This is equivalent to the dimension of love described in another model. And happiness and pain correspond to each other, which is equal to the dimension of love in the model. The policies and regulations related to corporate philanthropy can be divided into two categories: one is the normative and guiding policies for enterprises, and the other is the encouraging policies. Captivating spaces allow us to quantify changes and differences in people's psychological states. However, for further research on mental states, the two-dimensional mental state model cannot support deeper psychological research. Therefore, based on the two-dimensional mental model, it began to study three-dimensional and even multidimensional mental models, including Plutchik. Tension means that each mental state has a different tension. The same representative has different mental states under the same feeling. The stronger the two diametrically opposite polar states of mind, the stronger the dependence on their status. On the other hand, the weaker the state of mind, the lower its status, and the lower the state of mind. A state of bipolar manifestation is a diagonally similar form in a position next to the mental state. The occurrence, development, and results of human social events are the result of the interaction and joint action between the “socialized individual” and the objective external world.

RETRACTED

### 3.8. Definition and Calculation Characteristics of Big Data

Although a large number of researchers have conducted extensive and in-depth research on the idea of arrogant data since it was put forward, there is no precise definition so far. Many research institutions and scholars have determined a huge amount of data according to their own understanding, but these are only qualitative descriptions. Wikipedia defines big data as a group of data that cannot be obtained, which is managed and processed at a specific time using traditional and widely used software technologies and tools. The definition given by others is as follows: big data refers to a kind of transaction in which the size of the data set exceeds the possibility of acquisition, storage, and the management and analysis of traditional database tools.

The key characteristics of big data put forward new requirements and challenges for data processing and data mining. The data object processed by traditional data processing technology is structured data, which only represents a small part of the real data, and more than four-fifths of the data are semistructured or unstructured data, such as text or video. Traditional data processing techniques are powerless. Considering the above problems, in order to process big data efficiently, it is necessary to summarize different processing requirements and calculation characteristics according to different application characteristics.

## 4. Mental State Change Experiment

### 4.1. Experiment Content

This study selects “charity” in Baidu Tieba as an example and uses the crawler tool Python to collect data. It crawls a total of 17,818 floors of netizens' messages from December 4th to December 10th and uses this as the total sample. Through the method of equidistant sampling, 300 netizens' messages were selected as samples for content analysis. In these 17,818 floors, there is a lot of post-blogging phenomenon. During sampling, if the same brush post information is selected, the next one will be automatically selected, and so on, as shown in Figure 5.

RETRACTED

It can be seen that the search rates for the two terms, that is, charity activities for the disabled and charity activities for business personnel, are 17.3% and 16.6%, respectively. Charitable activities in these two areas are searched more frequently.

Table 1 is a cross-tabulation of the utterance types of the experimental subject platform.

A cross-sectional analysis shows that news information is the most published information by accredited organizations. This is also related to the fact that most of the publishing bodies are news organizations. Weibo big V publishes less knowledge and news information. Comments have the most information, with nearly half of them. Mobilization information accounted for more than one-third. The number of basic-level ordinary user comments and mobilization categories is equal.

It collects feature factors and builds models. Our model has a total of 6 reflective constructs and 21 items. The factor loading value of each item is examined, and all are greater than 0.7, so there is no need to process the item, and the final model will retain all the items as shown in Table 2.

As shown in the table, the combined reliability values for all constructs are greater than 0.7. Therefore, the credibility of the construct is considered to be high. In addition, the AVE values of all constructs were greater than 0.5, so the constructs were considered to have good convergent validity.

The intrinsic correlation coefficient of the latent variable shows the intrinsic correlation coefficient of the latent variables. The square root of AVE of a construct is greater than the correlation coefficient between this construct and other constructs, as shown in Table 3.

The correlation coefficients between constructs were all less than 0.7, and all were less than the square root of AVE. Therefore, it is considered to have good discriminant validity.

The PLS loads and cross loads are shown in Table 4.

It analyzes the communicative power of textual discourse. The forwarding and likes of each message are counted, so as to obtain the maximum, minimum, and average of the forwarding and likes in each type of discourse topic. In this way, the dissemination and influence of discourses on different topics are analyzed, as shown in Table 5.

It can be seen that the two discourse topics of “Charity Gala” and “Guarantee for the Disabled” are higher than the two discourse topics of “Charity” and “Analysis of Charity Forms” in terms of forwarding and likes. It shows that the discourse power and influence of these two aspects are more prominent.

RETRACTED

### 4.2. Development of Charity

With the development of philanthropy in China, public awareness of public welfare has been continuously enhanced. People have independently participated in charity activities through various channels, showing great enthusiasm for donation.  Figure 6 shows the amount of charitable donations in China from 2017 to 2021.

The data in the “2021 China Charitable Donation Report” shows that, in addition to a slight decrease in the total amount of charitable donations in 2018, the total amount of donations from 2017 to 2021 showed a steady upward trend as a whole. Especially in 2021, China's actual domestic and foreign donations (including cash and materials) will be 110.857 billion Yuan, accounting for 0.16% of the annual GDP, and the per capita donation will reach 8.169 billion yuan.

Figure 7 shows the donations received by various types of entities in 2021.

As can be seen from the figure, the foundation received donations of 44.557 billion Yuan, accounting for 40.19%. Charitable organizations received donations of 32.647 billion Yuan, accounting for 30%. Foundations and charitable organizations have become the two most important channels for donations, accounting for more than 70% of the total.

Figure 8 shows the proportion of corporate donations in 2019–2021.

It can be seen from the figure that corporate donations are still the most important source of social donations. This shows that enterprises have become an important force in promoting China's philanthropy.

### 4.3. Questionnaire Validity Test

Psychometrics believes that the correlation between each dimension and the total scale score exceeds the correlation between dimensions as a manifestation of construct validity. The mental health scale using social media attention to charity was sampled here. It examines the content validity of the questionnaire based on the correlation between each subscale and the total scale, as shown in Table 6.

The correlation between the questionnaire subdivisions and the overall scale ranged from 0.470 to 0.820. The correlation between dimensions is between 0.183 and 0.590. The correlation between each dimension and the total scale score is higher than the correlation between dimensions. This shows that the dimensions of the two scales are both related and different, and they are relatively independent and have certain construct validity.

It explores the proportion of male and female users of social media in a sample and conducts psychological research on philanthropy-based cultural behavior. The specific performance is to count the parameter matrices of all male and female users separately and make a graph comparison of 10 factors from A to J. The results are then compared, as shown in Figure 9.

RETRACTED

As can be seen from the figure, except for the factor A, the male data is much higher than that of females, and there is no significant difference in other items.

The more reference mental state changes can be discussed with the hierarchical affective model. The measurement of the basic emotional points of the PAD mood space is determined by psychological methods. Many researchers hope to reveal the location of basic emotions in the PAD space through research and experiments. By calculating the emotional distance between the unknown emotional point and each basic emotional point in the three-dimensional space of PAD mood, the basic emotion with the shortest emotional distance is selected as the emotional state of the unknown emotional point. In this way, the distance value between the unknown emotional point and each basic emotional point is obtained, as shown in Figure 10.

It can be seen from Figure 10 that the three items of PAD almost overlap in the emotional points from 1 to 10, while in the latter 5 points, they show a scattered form. This shows that when the emotional data set is very large, the PAD vector value of each basic emotional point tends to be stable, and the coordinate distribution in the PAD mood space is also relatively stable.

## 5. Discussion

### 5.1. Concept and Connotation of Charity Culture

Domestic scholars have done a lot of research on the topic of “charity culture,” and there are different opinions on its definition. In the research on the development of Chinese philanthropy, experts believe that philanthropy culture is knowledge and attitude. It is the feeling and evaluation of a country's philanthropy formed in the historical development. It is an important part of national culture and social culture. Among the different kinds of charity activities held on TV, the charity party can usually raise a large amount of money in a short time, and the effect is remarkable.

To understand the cultural construction of charity gala, we must deeply understand how the cultural connotation is manifested through different symbols in such a grand “media ceremony” as charity gala. A positive and healthy philanthropy culture has a positive effect on promoting philanthropy in a country. Philanthropic culture is functionally rich, but at its core are altruistic values. Charity culture is an important part of Chinese traditional culture. For centuries, China has emphasized philanthropy and poverty alleviation. It believes that people should pay attention to their own life and development and have a kind heart. People should recognize the social value of devotion and fraternity, deal with the difficult and needy people in society, express kindness and love within their ability, and provide help within their ability. Under the influence of a culture of charity, it promotes the creation of a “helping” social environment and the improvement of interpersonal relationships. Building bridges of communication and communication between members of society can bring people closer to each other. It is easy to eliminate the rigid and unfamiliar interpersonal relationships and the estrangement between different social classes when social audiences treat each other tolerantly. This has played a role in overcoming the growing social estrangement and promoting the development of a harmonious society.

RETRACTED

Charity and poverty alleviation have been traditional Chinese virtues since ancient times. The development of a philanthropic culture is inseparable from these traditional virtues. China's philanthropic culture has a long history and rich functions. Its development process can be roughly divided into three stages: the first is the ancient charity culture with “goodness” as the core, the second is the modern charity culture with the goal of “saving the country,” and the third is the modern charity culture with “human nature” as the core.

“Ritual view” pays attention to the maintenance of information on society in time. It does not mean the act of sharing information, but the representation of sharing faith. Therefore, it emphasizes not control and power, but sharing and communication. This definition reflects “Commonness,” “common,” “sharing,” and “communication.”

### 5.2. Theoretical Basis

#### 5.2.1. Social Action Theory

According to rationalism and degree of rationality, experts divide social behaviors into goal rationalization behaviors, value rationalization behaviors, emotional behaviors, and traditional behaviors. The expected rational action should demonstrate that the actor has a clear goal and understands the tools and means needed to achieve that goal. It is through expectations of external things and the behavior of others as conditions or means that they achieve their legitimate ends. The characteristic of rational value action is that it attaches great importance to the value of the action itself, regardless of the conditions required for taking the action and the consequences of the action. Essentially, the actor himself takes certain goals very seriously and is willing to hold on to their beliefs and uphold them. Emotional behaviors are behaviors that result from realistic emotions and emotional states. Emotions, on the other hand, relate to the social interactions the actor experiences and the subjective awareness of preexisting attitudes. Traditional movements are driven by habituation based on usual stimuli to repeat an established posture.

RETRACTED

In the process of charitable donation, enterprises can form a subtle force to affect all aspects of the enterprise. Through charitable donations, enterprises have established the social image of public welfare enterprises, accumulated corporate reputation, created a good external environment for the operation and development of enterprises, and promoted the improvement of enterprise performance.

It can be said that companies must meet consumers' expectations for more responsibility and create a positive image for increasing market share, thereby maximizing their own interests. Philanthropy is only the way and means for enterprises to realize their own interests. Explanations of corporate philanthropy with rational values tend to lean toward individual beliefs about the value of business owners or managers, or the expansion of corporate culture. This is the behavior of enterprises based on ethical pursuits. Some business owners or business managers encourage businesses to do charitable acts out of gratitude, empathy, or other feelings, based on their previous interactions or current stimuli. Obviously, emotional behavior is volatile and unpredictable. Using traditional behavior to explain corporate charitable behavior, corporate charitable behavior can be regarded as related to the social content accepted by corporate managers or related to the company's consistent corporate culture.

#### 5.2.2. Social Exchange Theory

From an economic point of view, corporate philanthropy is an act that indirectly promotes the maximization of interests. Interests here refer not only to economic interests, but also to political interests. Entrepreneurs share the pressure of the government in some functions through corporate philanthropy, so the government has a good impression of the enterprise. Business owners can obtain certain political recognition, thereby creating a favorable political environment for the business. Entrepreneur's political status allows companies to reduce the risk of acquisitions and ensure sustainable business development when they obtain certain basic resources controlled by the government. When this mutually beneficial relationship is established, businesses tend to become more involved in philanthropy. In addition, some scholars believe that corporate philanthropy is a defense mechanism for corporate crisis events and can accumulate moral capital for companies. When an accident happens to a business that negatively affects its image and reputation, charities can compensate or reduce the negative impact to a certain extent. Businesses are actively fulfilling their social responsibilities to avoid rational regulation. Because in the market competition, some business activities are regulated by the government. This regulation will reduce the company's profits and even force the company to cut production and stop production. When companies actively fulfill their social responsibilities and engage in charitable activities, they can basically avoid this regulation and improve their competitiveness in the market.

RETRACTED

## 6. Conclusions

In recent years, the explosive growth of data scale and the high complexity of data mode have prompted the current information society to enter the era of big data. In this era of rapid development, more and more people participate in charity. Charity culture is the driving force behind the development of philanthropy, and charitable culture also affects the development of philanthropy. Types of mental states are classified according to the level of mental activity. The level of positivity of mental activity is the internal cause of different mental states. It mainly refers to the degree of awakening and activity of the cerebral cortex, that is, the degree of awakening and activity of consciousness. Under such theoretical guidance and background significance, this paper selects “charity” in Baidu Tieba as an example. It collects data through the crawler tool Python, crawls a total of 17,818 floors of netizens' messages from December 4th to December 10th, and uses this as the total sample. Through the method of equidistant sampling, 300 netizens' messages were selected as samples for content analysis. It analyzes the amount of charitable donations in China from 2017 to 2021, as well as the donations received by various types of subjects in 2021, and draws a basic emotional PAD variance map in the sample. It analyzes the psychological state of other reasons for charitable cultural behavior and introduces the relevant content of social action theory and social exchange theory. It has well completed the subject of social media analysis and exploration of the psychological state changes of charitable cultural behaviors. In the follow-up research, more years of charitable donations should be selected as samples, and expanding the sample size can make the experimental results more authentic and reliable.

## Figures and Tables

**Figure 1:** Correspondence between text, latent variables, and terms.

**Figure 2:** Schematic diagram of the CBOW model.

**Figure 3:** Research pattern diagram.

**Figure 4:** Social media word-of-mouth research model.

RETRACTED

**Figure 5:** Cluster analysis of netizen message topics.

**Figure 6:** Charitable donations in China from 2017 to 2021.

**Figure 7:** Donations received by various types of entities in 2021.

**Figure 8:** Proportion of corporate donations in 2019–2021.

**Figure 9:** Comparison of gender differences in social media users based on charitable cultural behaviors.

**Figure 10:** Basic sentiment PAD variance plot in the sample.

**Table 1:** Discourse type cross tabulation.

	Knowledge class	News category	Comment class	Mobilization class	Total
Certification organization or institution	3	37	22	5	67
Certified individual	13	14	90	56	173
Ordinary grassroots users	0	4	17	15	36

**Table 2:** AVE, CR, and CA values.

	AVE	Cr	*α*
SP	0.8352	0.953	0.9342
MIC	0.786	0.9168	0.8662
EH	0.796	0.9397	0.9141
PC	0.8095	0.9271	0.8857
PR	0.6917	0.8703	0.7828
SW	0.7772	0.9331	0.9044

**Table 3:** Intrinsic correlation coefficients of latent variables.

	SP	Mic	Eh	PC	Pr	SW
SP	**0.9139**					
MIC	0.659	**0.8866**				
EH	0.6065	0.669	**0.8921**			
PC	0.0933	0.0283	0.0181	**0.8997**		
PR	−0.0351	−0.0434	0.0007	0.4328	**0.8316**	
SW	0.4991	0.5557	0.5864	−0.0949	−0.1049	**0.8816**

**Table 4:** PLS load and cross load.

	SP	Mic	Eh	*P*C	Pr	SW
SP1	0.8876	0.5965	0.5704	0.1497	−0.0498	0.4826
SP2	0.8825	0.5988	0.5318	0.0178	−0.061	0.472
SP3	0.9241	0.5988	0.5644	0.0892	−0.0072	0.4111
SP4	0.9332	0.6125	0.5488	0.0832	−0.0051	0.4501
MIC1	0.915	0.8826	0.6265	0.0383	−0.0577	0.5836
MIC2	0.5886	0.9116	0.5958	0.031	−0.0361	0.4414
MIC3	0.608	0.8651	**0.8239**	0.0005	−0.0142	0.4195
EH1	0.5527	0.5587	**0.9035**	0.0172	0.0602	0.452
EH2	0.4553	0.6013	**0.9275**	0.035	0.0093	0.511
EH3	0.5799	0.6286	**0.9103**	0.0105	−0.0111	0.5549
EH4	0.5891	0.589	0.0235	0.0039	−0.0433	0.565
PC1	0.5326	0.0295	−0.0116	**0.9132**	0.3834	−0.0776
PC2	0.0925	0.0374	0.062	**0.951**	0.3999	−0.1088
PC3	0.0904	−0.0023	0.0093	**0.8308**	0.3995	−0.055
PR1	0.0641	−0.0781	0.0232	0.4769	**0.7698**	−0.0821
PR2	0.0017	0.0112	−0.0176	0.3481	**0.8435**	−0.0555
PR3	−0.0054	0.0287	0.5383	0.2797	**0.8781**	−0.1081
SW1	−0.065	0.4956	0.4943	−0.1181	−0.0989	**0.8901**
SW2	0.4466	0.4549	0.4967	−0.0966	−0.0634	**0.8901**
SW3	0.4366	0.5042	0.535	−0.0183	−0.0865	**0.8733**
SW4	0.4571	0.5027	0.525	−0.0977	−0.1184	**0.8727**

**Table 5:** Transmission power analysis.

Topic	Maximum	Minimum forwarding volume	Mean value	Maximum	Minimum likes	Mean value
Charity party	209955	4	778.91	49353	4	2196.11
Philanthropic undertaking	16256	12	1502.81	74480	13	5918.81
Analyzing the form of charity	26752	4	871.16	66878	7	2059.6
Disability protection	50230	13	3122.97	94483	21	6192.97

**Table 6:** Correlation statistics of social media attention to charity mental health scale.

	F1	F2	F3	F4	F5	F6	F7	F8	F9	F10
F1	0.451^*∗∗*^									
F2	0.566^*∗∗*^	0.451^*∗∗*^								
F3	0,397^*∗∗*^	0.494^*∗∗*^	0.438^*∗∗*^							
F4	0.560^*∗∗*^	0.550^*∗∗*^	0.407^*∗∗*^	0.312^*∗∗*^						
F5	0.584^*∗∗*^	0.589^*∗∗*^	0.459^*∗∗*^	0.590^*∗∗*^	0.480^*∗∗*^					
F6	0.488^*∗∗*^	0.354^*∗∗*^	0.419^*∗∗*^	0.257^*∗∗*^	0.451^*∗∗*^	0.291^*∗∗*^				
F7	0.188^*∗∗*^	0.361^*∗∗*^	0.353^*∗∗*^	0.325^*∗∗*^	0.266^*∗∗*^	0.383^*∗∗*^	0.183			
F8	0.537^*∗∗*^	0.354^*∗∗*^	0.372^*∗∗*^	0.330^*∗∗*^	0.508^*∗∗*^	0.530^*∗∗*^	0.289^*∗∗*^	0.253^*∗*^		
F9	0.188	0.361^*∗∗*^	0.353^*∗∗*^	0.325^*∗∗*^	0.266^*∗∗*^	0.383^*∗∗*^	0.183	0.188	0.383^*∗∗*^	
F10	0.820^*∗∗*^	0.742^*∗∗*^	0.705^*∗∗*^	0.702^*∗∗*^	0.697^*∗∗*^	0.810^*∗∗*^	0.558^*∗∗*^	0.470^*∗∗*^	0.651^*∗∗*^	0.383^*∗∗*^

RETRACTED

## Data Availability

No data were used to support this study.

## References

[1] Rothkrantz L. (2017). How social media facilitate learning communities and peer groups around MOOCS. *International Journal of Human Capital and Information Technology Professionals*.

[2] Christian R. (2017). Towards social resilience: a quantitative and qualitative survey on citizens’ perception of social media in emergencies in Europe—ScienceDirect. *Technological Forecasting and Social Change*.

[3] Allcott H., Gentzkow M. (2017). Social media and fake news in the 2016 election. *The Journal of Economic Perspectives*.

[4] Enikolopov R., Petrova M., Sonin K. (2018). Social media and corruption. *American Economic Journal: Applied Economics*.

[5] Jeffery T., Monroe-Lord L., Ashe C., Bunchamroeun C. (2020). P32 evaluation of multilevel nutrition interventions among urban clients on charitable food assistance. *Journal of Nutrition Education and Behavior*.

[6] Sneddon J. N., Evers U., Lee J. A. (2020). Personal values and choice of charitable cause: an exploration of donors’ giving behavior. *Nonprofit and Voluntary Sector Quarterly*.

[7] Yang Y., Shi Y., Zhang D. (2020). Intergenerational effects on individual charitable donation: an innovative study on philanthropy in China. *Chinese Journal of Sociology*.

[8] Andreassen C. S., Pallesen S., Griffiths M. D. (2017). The relationship between addictive use of social media, narcissism, and self-esteem: findings from a large national survey. *Addictive Behaviors*.

[9] Khan M. L. (2017). Social media engagement: what motivates user participation and consumption on YouTube?. *Computers in Human Behavior*.

[10] Mnsted B., Sapieyński P., Ferrara E. (2017). Evidence of complex contagion of information in social media: an experiment using twitter bots. *PLoS One*.

[11] Ramanathan U., Subramanian N., Parrott G. (2017). Role of social media in retail network operations and marketing to enhance customer satisfaction. *International Journal of Operations and Production Management*.

RETRACTED

[12] Lee D., Hosanagar K., Nair H. S. (2018). Advertising content and consumer engagement on social media: evidence from facebook. *Management Science*.

[13] Bock D. E., Eastman J. K., Eastman K. L. (2018). Encouraging consumer charitable behavior: the impact of charitable motivations, gratitude, and materialism. *Journal of Business Ethics*.

[14] Heist H. D., Cnaan R. A. (2018). Price and agency effects on charitable giving behavior. *Journal of Behavioral and Experimental Economics*.

[15] Levens M. (2017). The influence of organic product classification on charitable contributions embedded in retail prices. *Economics and Culture*.

[16] Salonen A. S. (2017). Lining up for charity: a study of the social organization and communal qualities of breadlines in a Finnish city. *International Journal of Sociology and Social Policy*.

[17] Kim J. H., Seok B. I., Lee K. T., Yu J. P. (2017). Effects of social responsibility activities of franchise chain hotels on customer value and SNS citizenship behavior. *Journal of Franchise Management*.

[18] Gächter E., Renner E. (2018). Leaders as role models and ‘belief managers’ in social dilemmas. *Journal of Economic Behavior and Organization*.

[19] Krasnopevtseva V. V. (2017). Civic culture in contemporary Russia (on the example of Tula region). *Moscow State University Bulletin Series 18 Sociology and Political Science*.

[20] Kanukova Z. V., Tuaeva B. V. (2019). The Persian community in vladikavkaz: preserving ethnic identity in an alien cultural environment. *RUDN Journal of Russian History*.

